The article "Big Data Analysis of Manufacturing and Preclinical Studies of Nanodrug-Targeted Delivery Systems: A Literature Review" was retracted in 2023. Reasons: signs of a paper mill; unreliable results or conclusions; concerns about the data; concerns about the peer review.

# Big Data Analysis of Manufacturing and Preclinical Studies of Nanodrug-Targeted Delivery Systems: A Literature Review

**DOI:** 10.1155/2022/1231446

**Published:** 2022-07-30

**Authors:** Qiang Cao, Xiaochen Li, Qi Zhang, Kexuan Zhou, Ying Yu, Zixu He, Zhibiao Xiang, Yi Qiang, Wei Qi

**Affiliations:** ^1^School of Pharmacy, Macau University of Science and Technology, China; ^2^The Third Affiliated Hospital of Shandong First Medical University, China; ^3^Taishan University, China; ^4^Hainan University, China; ^5^University of New South Wales, University of New South Wales, Australia; ^6^Second Xiangya Hospital, The Second Xiangya Hospital, China; ^7^Kunming University of Science and Technology, China

## Abstract

**Objective:**

Nanodelivery is a modern technology involving improved delivery methods and drug formulations. The current development and initial applications of nanocarriers are pointing to new directions in the current development of nanomedicine. Researchers are increasingly applying nanodelivery to the delivery of therapeutic or diagnostic agents. This article discusses the preparation and application of nanocomplexes and nanoparticles, as well as their potential future value in clinical research. Through a review and analysis, it is hoped that this will serve as a guide for the future development of various nanodelivery technologies and help researchers learn more about these technologies.

**Materials and Methods:**

A literature search was conducted using the keywords “Nano drug delivery” or “Nanomedical materials” or “Nano”. A literature search was conducted in three major databases, PubMed, Web of Science, and Google Scholar, using the keywords such as “Nano drug delivery”, “Nanomedical materials”, or “Nanobubble drug delivery”. The initial search was screened by title and abstract. In the full-text review, the titles or abstracts were reviewed according to the selection criteria based on the inclusion criteria. The risk of bias and study quality was assessed according to the Cochrane guidelines, and possible biases such as selection bias and good selection bias were included in the review.

**Results:**

A total of 297 studies were included in this study, of which 219 were excluded based on the screening criteria, resulting in the inclusion of 78 studies, the majority of which were original studies and clinical trials, and a small number of which provided design and route of administration analysis of nanomaterial particles and effect fluorograms and were studied in more depth. This paper summarises and reviews the views and directions of the included articles. The main directions include cyclodextrin-based or grafted cyclodextrin nanomaterials, nanobubbles, and stimuli-sensitive and temperature-sensitive nanodelivery systems.

The article "Big Data Analysis of Manufacturing and Preclinical Studies of Nanodrug-Targeted Delivery Systems: A Literature Review" was retracted in 2023. Reasons: signs of a paper mill; unreliable results or conclusions; concerns about the data; concerns about the peer review.

**Conclusion:**

The use of innovative, targeted drug delivery systems is effective in cancer drug delivery by summarising the previous studies. However, nanodelivery systems' risks and therapeutic effects need to be evaluated before clinical application. Future research in the field of targeted drug delivery nanosystems should focus on the development of nanocarriers with high in vivo delivery capacity, good synergy with therapeutic agents, and milder short-term and long-term toxicological effects and conduct comprehensive preclinical trials on nanodrug delivery systems with high potential for clinical application as soon as possible, to find nanodrug delivery systems suitable for clinical use and put them into the clinical application as soon as possible.

## 1. Introduction

The materials chosen for nanodelivery can come from almost any substance, lipophilic colloidal nanoparticles (NPs) from solid lipids and phospholipids and nanomaterials based on carbon, natural, or synthetic polymers, and metal oxides can also be used. In bio-nanotechnology, nanomaterials are used in biomedical applications, including targeted drug delivery, contrast agents, and biosensors. Many nanomaterials' properties allow them to be used in drug delivery processes but can also make them toxic to living cells. Due to their large surface area, nanomaterials are more active and can easily cross environmental barriers, pass through cell membranes, and enter the body. In order to maximize the potential of nanotechnology, a sound scientific approach to nanotoxicology and safety issues is required. There are many different approaches in preparing NF, using both conventional and unconventional techniques in both the solid and liquid phases [1]. The main objective is to obtain NFs of uniform size and shape. Several techniques have addressed this issue; mechanochemistry is used in solvent-free solid-phase synthesis, while microwave radiation and ultrasonication are used for synthesis in aqueous solutions.

As a heat source with a high heating rate, microwave irradiation can produce large quantities of high-quality NS in a short period. The application of microwave irradiation allows for a high degree of homogeneous mixing of raw materials and reduced crystal production during the preparation of nanomaterials. It increases the reaction rate when preparing nanomaterials [2, 3]. Sonochemical and microwave-assisted synthesis development can be effectively applied to the derivatization of carbon-based nanomaterials and the production of nanostructured cyclodextrin oligomers and grafted nanomaterials for biomedical applications. Studies have shown that CD derivatives can retain drug and contrast agent molecules and be used as versatile and efficient carriers and contrast agents for MRI. Grafting CD onto NF can increase its water solubility and surface accessibility. Since the nanobubbles are spherical in structure, multifunctional nanocarriers can be developed on nanobubbles (core/shell) for targeted imaging and therapy. It has become increasingly important to improve the efficacy of antitumor drug nanosystems and to use nanodelivery strategies for successful treatment, as they enable “on-demand” drug release and tailored delivery regimens. In an ideal, it would be able to deliver the appropriate medication at the appropriate time to the appropriate patient.

The article "Big Data Analysis of Manufacturing and Preclinical Studies of Nanodrug-Targeted Delivery Systems: A Literature Review" was retracted in 2023. Reasons: signs of a paper mill; unreliable results or conclusions; concerns about the data; concerns about the peer review.

## 2. Methods

The current literature search was conducted using PubMed, Web of Science, and Google Scholar until 9 May 2022 with the following search terms: “Nano drug delivery” or “Nanomedical materials” or “Nanobubble drug delivery”, including original research, randomized trials, clinical trials, reports, and guidelines.

The articles were initially screened by title and abstract. The review of titles or abstracts against inclusion criteria was carried out in a full-text review based on selection criteria and assessed for risk of bias and study quality against Cochrane guidelines, with potential bias such as selection bias and good selection bias included in the review, with two members of this group dedicated to bias assessment and ultimately consensus within the group. After the bias assessment, exclusion of some literature that would pose a risk of bias to this study, the contents of the literature were put together, and the references in the literature were used to make a data network from which the data and discussion that would support this study were eventually gathered. This study is a review article conducted following the PRISMA-P statement and did not require approval by the ethics committee before proceeding with the study.

## 3. Results

After a search exercise in three databases, a total of 297 studies were included in this study, of which 219 were excluded based on the selection criteria, resulting in the inclusion of 78 studies, most of which were original studies and clinical trials, and a small number of which provided the design of nanomaterial particles with the route of administration analysis and effect fluorograms of and conducted more in-depth studies. Different members wrote two articles on the same unit or subject group, and their conclusions were similar. Some of the included articles have not been peer-reviewed. This poses a slight challenge to the research work in this paper. The relevance of the included literature is shown in Figure 1. This paper summarises and synthesizes the views and directions of the included articles. It focuses on the current status and prospects of intelligent nanosystems for drug delivery controlled by specific internal or external factors.

The article "Big Data Analysis of Manufacturing and Preclinical Studies of Nanodrug-Targeted Delivery Systems: A Literature Review" was retracted in 2023. Reasons: signs of a paper mill; unreliable results or conclusions; concerns about the data; concerns about the peer review.

### 3.1. Cyclodextrin-Based or Grafted Cyclodextrin Nanomaterials

The use of nanotechnology for drug delivery offers new opportunities for the delivery of therapeutic drugs to intracellular targets and monitoring target delivery sites, which could influence the future development of the pharmaceutical and biotechnology industries. In the future, nanodrug delivery systems may be able to achieve targets with good biocompatibility and improve the physicochemical properties of drugs (stability, solubility, and bioavailability) [4]. As with other synthetic methods, unconventional techniques using ultrasound and microwaves have been widely used to prepare new versus known structures based on CD, and in experiments, this approach has shown good efficiency and short reaction times. The production of a water-soluble phosphate oligonucleotide isomer by ultrasound as a dendritic multicarrier with high receptivity and its suitability as an MRI contrast agent has been successfully demonstrated in relaxation titration experiments of Gd complexes placed on a dendritic polymer platform and in successful experiments regarding cell viability and binding capacity [5–7]. Microwave radiation has currently been demonstrated to enable the derivatization of carbon nanotubes (SWCNTs) with CD and contrast agents [8, 9]. The effectiveness of microwave exposure has also been demonstrated for producing graphene oxide grafted to porphyrins [10]. With the help of these antecedent studies, it is currently possible to investigate the ability of CD to attach or release drugs concerning magnetic NPs. NFs of iron oxide and gold were obtained as a versatile nanodesign platform by attaching to a polyacetal methacrylate bound to CD and functionalized with ethylenediamine [11]. Under ultrasonic irradiation, the magnetic NFs were coated with *β*-cyclodextrin, increasing magnetization, possibly due to the high degree of crystallization of the resulting final material [12].

### 3.2. Development and Application of a Drug Delivery System with Nanobubbles

*Nanobubbles* are substances that are sensitive to external physical factors. Nanobubbles originate from microbubbles and are currently used as contrast agents in clinical practice. This characteristic determines several advantages, such as their ability to enter the surrounding tissue from the vasculature to improve imaging and targeted delivery. In particular, this ability allows them to accumulate in tumor tissue over time due to the effects of increased permeability and retention (EPR). Furthermore, ultrasound exposure enhances the acoustic and targeting properties of such nanobubbles so that nanobubbles can be used as therapeutic cavitation nuclei for ultrasound treatment, leading to the formation of temporary pores in the plasma membrane as altering cell permeability [13].

The article "Big Data Analysis of Manufacturing and Preclinical Studies of Nanodrug-Targeted Delivery Systems: A Literature Review" was retracted in 2023. Reasons: signs of a paper mill; unreliable results or conclusions; concerns about the data; concerns about the peer review.

Nanobubbles can be described as spherical structures with a core and a shell filled with gaseous or evaporative components such as perfluorocarbon, sulfur hexafluoride, air, or carbon dioxide [14]. The core region occupies most of the volume of the particle, and it can influence the structural and functional properties of the nanobubble. When there are no other influencing factors (such as charge), insoluble gas is surrounded by a liquid, the hydrophobic group reaches inside the bubble, and the hydrophilic group reaches into the liquid. Therefore, nanobubbles made of insoluble gases have lower surface tension than those made of other gases, which can ensure the stability of nanobubbles. This makes the nanobubbles stable and gives them a long life. Due to the compression/decompression cycles of ultrasound, the compressibility parameters of the gas core can significantly impact the volumetric fluctuations of the system. Fluctuations in the gas bubble volume can enhance echogenic backscatter and promote drug release, which can improve the effectiveness of diagnostic imaging and therapeutic applications, respectively.

The composition of the vesicle envelope determines its stiffness and resistance to degradation in ultrasound pressure fields, recognition by the reticuloendothelial system, and biodistribution [15]. The envelope is usually composed of lipids (phospholipids and cholesterol), polymers, polysaccharides, or proteins. These include nanobubbles with a perfluorocarbon core and a polysaccharide shell; their use has shown exciting results [16]. These are hybrid polymer-lipid systems developed to address the stability issues of nanobubbles and improve drug binding capabilities. The presence of polysaccharide shells allows for interaction with specific ligands.

Table 1 shows a list of biomolecules that enter the perfluorocarbon polysaccharide nanobubbles differently. The hybrid system contains a monolayer of phospholipids that can interact with polyelectrolytes. The structure of this hybrid lipid-polymer system is based on the fact that the phospholipid monolayer can adsorb charged polymers, such as polysaccharides, through various types of interactions, including electrostatic hydrophobic. Attempts have been made to create smaller nanobubbles. Most of these involve technical manipulation of the microbubbles during preparation, such as gravity gradient separation, physical filtration, or flotation. An alternative approach to achieving this goal is the initial formation of nanoscale systems. Nanobubbles are obtained mainly by ultrasonic treatment, high shear emulsification, thin layer evaporation, and mechanical stirring; these procedures are also used to obtain microbubbles [13]. Nanobubbles are a versatile tool for developing externally controlled nanocarriers with the controlled release of active drugs and imaging capabilities. Nanobubbles show high drug binding (encapsulation) efficiency and prolonged drug release.

The article "Big Data Analysis of Manufacturing and Preclinical Studies of Nanodrug-Targeted Delivery Systems: A Literature Review" was retracted in 2023. Reasons: signs of a paper mill; unreliable results or conclusions; concerns about the data; concerns about the peer review.

### 3.3. Stimulation-Sensitive Nanosystems

The effectiveness of drug therapy depends mainly on how the active ingredient reaches the target organs and tissues. On the way to the target, drug molecules can be affected by enzymes and have problems accessing the target area and cell selectivity. In this regard, the development of targeted drug delivery systems utilizing LF holds great promise for applications, with both passive and active targeting showing promising results. In addition, the novel properties of such nanosystems have the potential to enhance the bioavailability of drugs at the desired site. Targeted drug delivery systems for PM ensure that the drug leaves the bloodstream only at the target site or “target organ,” where passive or active PM accumulation occurs. The use of low-density drug delivery ensures better access to specific organs and prevents the elimination of drugs due to first-pass effects in the liver. Passive accumulation occurs due to the EPR effect observed in pathological tissues. For example, in tumor cells, NF accumulation is much faster than in other tissues and is characterized by uneven distribution and particle size dependence. Accumulation of activity is achieved due to specific interactions of the nanosystem with the target cells—due to the presence of monoclonal antibodies or bioconjugates on the NS surface [17]. However, NF's targeted drug delivery systems are often accompanied by systemic side effects associated with nonspecific biodistribution and uncontrolled drug release patterns. Several nanoformulations for cancer treatment have been proposed in the pharmaceutical market, and they have shown a better safety profile than conventional drugs. However, researchers have noted low bioavailability of drugs within the tumor and insufficient therapeutic efficacy [18]. Researchers in related fields are currently seeking modern nanodelivery systems that enable controlled drug release in space and time to overcome these problems. Joint developments in nanomaterials and pharmaceutical research are paving the way for the development of innovative nanodelivery systems, particularly in the treatment of cancer, where nanomaterials can play a therapeutic role together with drugs. Intelligent nanosystems that are sensitive to external or internal factors can improve drug efficacy and reduce side effects, resulting in intelligent stimulus-sensitive nanosystems [19].

The article "Big Data Analysis of Manufacturing and Preclinical Studies of Nanodrug-Targeted Delivery Systems: A Literature Review" was retracted in 2023. Reasons: signs of a paper mill; unreliable results or conclusions; concerns about the data; concerns about the peer review.

There are two types of stimulus-sensitive nanosystems available, i.e., nanodelivery systems that can respond to changes in the biological environment and thus regulate the rate of drug release based on a feedback system and delivery systems that can activate and release a drug in response to some external trigger. In both systems, sensitivity to internal or external stimuli can be achieved by using nanomaterials carrying functional groups that can change their properties depending on the strength of the signal. This leads to changes in the properties of the nanosystem, such as the ability to release the drug. These changes may have different properties, but a nanodelivery system can only be considered intelligent if these structural changes are reversible and proportional to the intensity of the stimulus [18].

### 3.4. Nanosystems Sensitive to Internal Stimuli

#### 3.4.1. Nanoparticles with Redox-Dependent Reactions

The design and development of NFs with a redox response are another direction for targeted drug delivery to specific sites within tumor cells. Glutathione oxidation systems that have entered clinical trials are being used initially in cancer cell therapy and have been selected as a reference model for developing redox-dependent nanocarriers. It has been shown that the concentration of glutathione localized in tumor cells is 100-500 times higher than in normal cells [19–23]. GSH levels in the intercellular space may cause bond exchange in the thiol-disulfide system. Polymers with disulfide bonds in their structure can successfully exploit this property to release drugs rapidly in response to glutathione stimulation. There are two ways to exploit the properties of disulfide bonds in polymer systems, i.e., modifying disulfide bonds directly on the polymer framework versus creating disulfide bonds in the polymer network as a cross-linking agent.

A 2019 study suggested improvements to active ingredient delivery systems, suggesting that glutathione-sensitive nanofibres that are unstable inside cells could be used [24]. The disulfide bonds of polymers can maintain their stability in the extracellular space for long periods but lose their stability once inside the cell. As a result, the bioavailability and efficiency of redox-dependent nanosystems are improved. The depletion of endogenous antioxidants makes cancer cells more susceptible to chemotherapeutic agents. This research has driven the generation of a new class of glutathione-sensitive CD nanodelivery systems designed to deliver doxorubicin in a targeted manner to cells with high GSH content. Glutathione-specific carriers loaded with doxorubicin inhibited clonal growth, cell viability, and enzyme activity and induced more structural DNA damage than other delivery methods when observed in different cell lines. Notably, the use of this system inhibited prostate tumor development more effectively than the administration of unconjugated drugs, without additional toxicity. Due to the nanosystem's precise delivery, doxorubicin can act more specifically on cancer cells and less on healthy cells near the cancer cells. This means that doxorubicin delivered by the nanosystem has less of an effect on healthy cells than free doxorubicin, ensuring therapeutic efficacy and minimizing side effects.

The article "Big Data Analysis of Manufacturing and Preclinical Studies of Nanodrug-Targeted Delivery Systems: A Literature Review" was retracted in 2023. Reasons: signs of a paper mill; unreliable results or conclusions; concerns about the data; concerns about the peer review.

#### 3.4.2. Reaction of Nanoparticles with pH Dependence

A typical example of a stimulus-dependent nanosystem that responds to internal signals is the operation of pH-sensitive nanocarriers for targeted transport to dense tumors. Low pH in the extracellular matrix caused by glycolytic activity in tumor tissue can be a specific stimulus for the nanosystem. Given that surface potential is directly related to cellular uptake, charge-induced polymeric nanosystems have been proposed for targeted delivery to tumor tissue. Positively charged NF exhibits good permeability due to positive interaction with the cell membrane. Furthermore, this NS can act like a “proton sponge,” causing disruption of lysosomes, facilitating intracytoplasmic delivery, and inducing cancer cell death [20]. The new tetrasaccharide-based polymer obtained by Caldera et al. is a chain of cyclic nigrosugar-1-6-nigrosugar (CNN). Cross-linking the four glucose and caramel dihydrates produced the entire NF described as “nanoporous” (NG). The polymer was characterized by its biocompatibility and ability to be selectively assimilated by cells according to pH changes. Doxorubicin is well encapsulated in the nanostructure and shows a slow and stable release pattern. The combination of the pH specificity of doxorubicin and the prolonged release capacity in the CNN nanostructures, which enhanced the antitumor effect, suggests the success of this nanostructure as a nanomedical tool while showing a milder toxicological profile and common side effects of the therapy [21].

The pH-dependent blocking of SiO_2_ mesopores using fluorescently labeled CD derivatives has also demonstrated favorable release kinetics of doxorubicin. The ability to monitor the movement of fluorescently stained NPs during treatment provides an advantage for applying this substance [22].

The article "Big Data Analysis of Manufacturing and Preclinical Studies of Nanodrug-Targeted Delivery Systems: A Literature Review" was retracted in 2023. Reasons: signs of a paper mill; unreliable results or conclusions; concerns about the data; concerns about the peer review.

### 3.5. Nanosystems Sensitive to External Stimuli

#### 3.5.1. Nanoparticles Sensitive to Temperature and Ultrasound

Controlling the rate of drug release from the nanocarrier by temperature changes is the most common way of delivering drugs. Under pathological conditions, for example, the temperature of cancerous tissue is higher than the temperature of healthy tissue. This difference can act as a trigger for releasing the drug at the tumor site. Thermosensitive nanocarriers are designed to not release the drug formulation at physiological temperatures (37°C) and to release the drug when the temperature rises to 40-45°C. For safety reasons, the temperature range of most nanocarriers is calculated so that the threshold of sensitivity to temperature signals exceeds the background temperature fluctuations. By combining the effects of thermotherapy in the presence of temperature-sensitive liposomes, a specific release of the drug substance in the tumor can be achieved.

#### 3.5.2. Nanoparticles and Nanobubbles Sensitive to Ultrasound

Ultrasound is widely used in clinical diagnosis and treatment, mainly due to its high penetrating power and safety for the body. Low-frequency ultrasound can penetrate body organs and act on body tissues and organs in various ways including local temperature elevation. The effect depends on the frequency of the waveband used, the intensity of the radiation, and the duration of the exposure. Local heating of tissues with ultrasound is widely used in clinical practice (focused high-intensity ultrasound), while the therapeutic effects of nonthermal ultrasound irradiation have been less studied. In addition to thermal effects, ultrasound is also used to convert the permeability of biological barriers and regulate drug delivery; it is used in ultrasound therapy.

Sonodynamic therapy (SRT) is a technique in which low toxicity molecules are activated by physical exposure to ultrasound, leading to oxidation, damage, and death of cancer cells. The effects of SRT are achieved by applying an external stimulus in the presence of the molecules or colloidal systems activated by it. The combination of these two factors, in turn, provides a biological effect. Acoustic cavitation is the formation or operation of a cavity filled with gas or vapor (bubbles) in a medium subjected to ultrasonic action. Two states of acoustic cavitation are distinguished.

A steady state in which oscillations cause the liquid to evaporate and mix with the surrounding microenvironment

Inertial state in which the growing cavity will grow to the maximum volume attainable at the ultrasonic wavelength in which it is located, producing an explosion upon reaching its maximum value. In the second case, the temperature of the microenvironment surrounding the explosion may rise sharply to 10 000°C, and the pressure may reach up to 81 MPa, turning the system into a kind of “acoustic-chemical reactor” [25]. In anticancer therapy, LF can be used as a stimulus-dependent acoustic sensitizer with improved spatial and velocity properties and as an acoustic sensitizer in its own right if cleverly designed [26]

The significant anticancer activity of polymethylmethacrylate containing 4-sulfophenyl porphyrins was demonstrated in an in vitro neuroblastoma model when the target site was exposed to ultrasound [27, 28]. These NFs can act as acoustically sensitive systems for in vivo applications, as radiolabelling and magnetic resonance imaging agents, and their suitability for targeted therapy and imaging of dense tumors. The nanosystems were loaded with 4-sulfophenyl porphyrin for anticancer or 64Cu-TPPS for diffusion topography studies in positron emission tomography. Based on a comparison of MR data taken before and after treatment in a synthetic breast cancer model, the TPPS-RMANCH nanosystem showed sensitivity to ultrasound. The 4-sulfophenyl porphyrin and polymethyl methacrylate carried by the TPPS-RMANCH nanosystem can work as an anticancer agent in ultrasound therapy by combining their effects, suggesting that this multimodal system could be successfully used as a selective external control tool for cancer control [29].

The article "Big Data Analysis of Manufacturing and Preclinical Studies of Nanodrug-Targeted Delivery Systems: A Literature Review" was retracted in 2023. Reasons: signs of a paper mill; unreliable results or conclusions; concerns about the data; concerns about the peer review.

In order to better understand the unique properties of inorganic NPs and, in this case, gold, the properties of gold have also been investigated to understand its LPR phenomenon better. NF made from gold coupled to folic acid polyethylene glycol has been shown to act as an adjuvant sensitizer for cancer treatment. Sensitivity to ultrasound exposure was studied on human cancer cell lines with varying numbers of folate receptors. Gold-made NF was selectively sensitive to folate receptors in highly expressed cancer cells, leading to decreased cell growth, increased production of reactive oxygen species, and increased necrotic cells through ultrasound exposure [30]. Exploiting the synergy between the precise targeting of gold NF and the sensitizing effect obtained through local external stimulation could make the nanosystem a promising platform for site-specific cancer treatment. This in vitro study can be considered as evidence that gold nanofibres have the potential to be used in the treatment of cancer.

The article "Big Data Analysis of Manufacturing and Preclinical Studies of Nanodrug-Targeted Delivery Systems: A Literature Review" was retracted in 2023. Reasons: signs of a paper mill; unreliable results or conclusions; concerns about the data; concerns about the peer review.

One study investigated the feasibility of combining nanobubbles with ultrasound irradiation for the topical treatment of dermatological conditions. A vehicle was developed to treat localized skin lesions associated with hypoxia while accelerating wound healing [31, 32]. That study also developed decafluoropentane- or dodecafluoropentane-loaded nanobubbles with dextran and chitosan shells for oxygen delivery, capable of dissolving and storing oxygen in their cores and releasing it slowly and stably due to their perfluorocarbon properties [32–35]. Under both in vitro and in vivo conditions, the decafluoropentane system showed significant efficacy in delivering oxygen to hypoxic regions, as evidenced by comparative analysis using oximetry and photoacoustic imaging. By exploiting the antimicrobial properties of chitosan, oxygen-loaded nanodroplets in chitosan shells have been proposed as an innovative tool to aid in treating infections in patients with chronic skin diseases [32, 36]. Oxygen-loaded nanodroplets exhibited high cytostatic activity against methicillin-resistant Staphylococcus aureus (MRSA) and Candida albicans, with no toxic effect on human keratinocytes (HaCaT). In addition, additional ultrasound exposure promoted transdermal delivery of oxygen from nanodroplets to tissues exposed to hypoxia. Research in recent years has focused on an in-depth study of the morphology of nanobubbles that facilitate oxygen transport, as exogenous oxygen delivery to tumors is difficult if removed from the bloodstream. The excellent solubility of oxygen in the bubbles gives them an advantage in delivering oxygen to hypoxic tissues.

Nanobubbles made of dextran sulfate were designed for targeted drug delivery in skin infections [37]. The combined use of targeted drug delivery and ultrasound irradiation facilitated the penetration of antibiotics into the skin through the action of ultrasound electrophoresis, and targeted drug release occurred at the site of disease.

Diethylaminoethyl dextran (DEAE) nanobubbles have been applied to protect proteases and the transport of DNA molecules loaded therein for plasmid DNA transfection across cell membranes. No cytotoxic effects were observed in this case [38]. Another chitosan-based nanobubble formulation has been proposed for the transport of DNA. The nanobubbles containing DNA have dimensions of up to 300 nm while accommodating a considerable amount of DNA [39]. In vitro transfection experiments were also performed. Adherent cells of the COS7 line were exposed to ultrasound at a frequency of 2.5 MHz in the presence of different concentrations of nanobubbles filled with plasmid DNA. None of the transfections were successful without ultrasound stimulation in all concentrations tested. Thirty seconds of ultrasound exposure showed a moderate success rate of transfection. Cell viability studies showed that neither ultrasound nor nanobubbles adversely affected the system under the experimental conditions performed.

The article "Big Data Analysis of Manufacturing and Preclinical Studies of Nanodrug-Targeted Delivery Systems: A Literature Review" was retracted in 2023. Reasons: signs of a paper mill; unreliable results or conclusions; concerns about the data; concerns about the peer review.

In recent years, the ongoing efforts of cancer immunotherapy researchers have led to several vaccination concepts based on tumor-associated antigens, such as the oncogene HER2. Anticancer vaccination offers several distinct advantages over standard therapies. These include higher specificity, lower toxicity, and gentler long-term effects caused by immune memory. In this sense, nanotechnology has great potential to improve the quality of immunotherapy significantly. After all, to qualitatively improve the immune response to tumor development, the vaccine must first reach the relevant dendritic cells, which play a crucial role in inducing the correct immune response. In recent years, a novel immunotherapeutic tool, namely, chitosan nanobubbles carrying a DNA vaccine and equipped with anti-CD11C surface antibodies for targeting dendritic cell recognition, has been developed for the treatment of HER2-positive breast cancer [40]. Subcutaneous injection of pHER2-loaded CD11c nanobubbles exhibited migration of skin dendritic cells to excretory lymph nodes and inhibited the growth of HER2-positive tumors. Therefore, researchers are investigating various modifications of nanobubbles as a diagnostic-therapeutic platform to exploit their echogenic properties. Polymeric nanobubbles are a versatile tool for targeting cancer cells, ultrasound imaging, and performing ultrasound-guided cancer therapy.

UK researchers have developed a variant of chitosan nanobubbles as a diagnostic-therapeutic system capable of dual visual detection of nanobubbles [41]. A variant of this nanosystem simultaneously delivers prednisolone phosphate, placed at the leading edge of a perfluorobutane core, and electrostatically binds the negatively charged GD-DOTP complex to a cationic chitosan body. The nanobubbles exhibited echogenic properties, which allowed them to be used in real-time imaging systems while showing positive contrast in magnetic resonance studies. The effects of extracorporeal shock waves (ESPs) were investigated as another external stimulus to which the response (in addition to ultrasound) may lead to the release of the active components of the nanosystem. EUV is a brief (less than 10 ms) focused acoustic oscillation widely used in urology for lithotripsy and the treatment of various motor dysfunctions. The efficacy of nanotransport bubbles under EUV stimulation has been extensively studied. Notably, the efficacy of the combined action of nanobubbles and UV light has been studied in at least two aggressive cancers, asexual thyroid cancer and prostate cancer [42–45]. Cotreatment with nanobubbles loaded with paclitaxel or docetaxel and EBV has been reported to increase the cytotoxicity of both drugs in two prostate cancer cell lines (PC3 and DU145). This study reduced the GI50 dose of paclitaxel to 55% and docetaxel to 45% (Figure 2).

The article "Big Data Analysis of Manufacturing and Preclinical Studies of Nanodrug-Targeted Delivery Systems: A Literature Review" was retracted in 2023. Reasons: signs of a paper mill; unreliable results or conclusions; concerns about the data; concerns about the peer review.

#### 3.5.3. Nanoparticles with Light-Dependent Reactions

Drug release from light-dependent nanosystems is triggered by exposing the particles to a specific wavelength of light from an external source. However, the low light penetration makes such systems extremely limited in their application. In light-dependent nanodelivery systems, the drug can be bound to a carrier through photodegradation bonds or by a carrier that can change its structure under specific light exposure. The infrared light-dependent resetting effect of doxorubicin, for example, was demonstrated by a matrix made of a lactic acid polymer with a coating [46, 47]. Gold-containing drug delivery nanosystems have attracted more attention in academia due to their ease of fabrication and good biocompatibility. Such NFs can be used as targets for local plasmon resonance, a technique used in multimodal cancer therapy, particularly in photothermal therapy [48]. Under near-infrared irradiation, gold-containing low-frequency resonances lead to local heating (several degrees above body temperature values). After intravenous injection, these NFs are exposed to a laser brought in by a fiber optic, which initiates local heating at the tumor nodes, thus providing photothermal therapy [49]. In addition, the surface of gold-containing NFs is suitable for attaching drugs, oligonucleotides, and peptides [50, 51]. Such nanoparticles can be successfully applied for targeted substance delivery and release tasks under the influence of external signals [52].

## 4. Discussion

In recent years, research trends in nanoparticle drug delivery systems have fully reflected the interdisciplinary cross-fertilization, synergy, and innovation between biologists, chemists, and clinical researchers. Targeted drug delivery systems based on nanoparticles provide better technical support for clinical disease treatment research. As a new and popular drug delivery system, nanocarriers have excelled in targeted therapy and tumor diagnosis and delivery. However, issues related to potential toxicity, accurate targeting of deep lesions, and true efficacy still need to be addressed. Only a few nanodelivery systems are currently in clinical trials. Most studies are still in the experimental stage. The large-scale clinical application of nanodelivery systems is limited by many factors, including drug release performance, optimization of the preparation process, production costs, surface properties of nanosystems, and in-depth studies of in vivo mechanisms of action. As the design of research nanosystems is optimized and research continues, however, nanodelivery systems are gradually overcoming their inherent limitations and providing more options for the development of new, safe, and effective nanoparticle drug delivery systems.

The article "Big Data Analysis of Manufacturing and Preclinical Studies of Nanodrug-Targeted Delivery Systems: A Literature Review" was retracted in 2023. Reasons: signs of a paper mill; unreliable results or conclusions; concerns about the data; concerns about the peer review.

Compared to drug or gene therapy alone, nanodelivery systems combine nanotechnology and targeted drug delivery technologies. By combining the two different mechanisms of action, the synergistic effect can be improved, and drug tolerance, for example, in tumor cells, can be reduced. The exact intracellular delivery mechanism for drug delivery by nanoparticles is still unclear from the current research. To investigate how to ensure optimal synergy between the drug and the nanodelivery system when the drug is loaded onto the nanoparticles remains. In addition, although nanoparticles can carry and deliver drugs in vivo with relatively mild short-term toxicological effects, their potential long-term toxicity in the body needs to be further investigated and their metabolic pathways and clearance mechanisms. The ideal vehicle should be able to deliver the drug with a good delivery capacity. However, it should also be able to precisely regulate the site, time, and dose of release to achieve the maximum effect of the combination therapy. Further research should focus on the synergy between the therapeutic agent and the carrier.

With the rapid development of nanotechnology and related research, targeted drug delivery systems based on combined therapy have more advantages than single function and composition drug delivery systems in ultrasound therapy and tumor delivery. Nanodelivery systems have shown promising applications, and research on ultrasound therapy and precision killing of cancer cells will hopefully make further progress in the continuous development of nanodelivery systems.

## 5. Conclusion

A review of previous studies demonstrates that intelligent, targeted drug delivery systems are highly effective for the delivery of anticancer drugs. Prior to their use in clinical applications, however, a comprehensive assessment of their therapeutic efficacy and potential risks is required. Future research in targeted drug delivery nanosystems should focus on the development of nanocarriers with high in vivo delivery capacity, good synergy with therapeutic agents, and milder short-term and long-term toxicological effects to enhance the clinical benefits of nanodrug delivery systems. Researchers should continue to refine nanodelivery systems and conduct thorough preclinical trials on those with a high potential for clinical application to find suitable nanodelivery systems for clinical use and put them into clinical use as soon as possible.

The article "Big Data Analysis of Manufacturing and Preclinical Studies of Nanodrug-Targeted Delivery Systems: A Literature Review" was retracted in 2023. Reasons: signs of a paper mill; unreliable results or conclusions; concerns about the data; concerns about the peer review.

## Figures and Tables

**Figure 1:** Searching for “Nano drug delivery”, “Nanomedical materials”, or “Nano bubble drug delivery” as keywords and summarising the literature resulted in a literature association chart.

**Figure 2:** Fluorescence intensity of DU145 (a) with PC3 (b) treated with 6-coumarin-labelled glycol chitosan NBs (15-104 NBs/ml) for 24 hours. Quantitative analysis of 6-coumarin-labeled glycol chitosan NBs in DU145 (c) and PC3 (d) cells and significance of DU145 (c) compared to 6-coumarin-labeled glycol chitosan NBs and no ESWs in PC3 (d) cells.

**Table 1:** The case of nanobubble delivery of bioactive substances.

Treatment effects	Medicinal product	Method of administration
Diagnostic systems	Gd complexes	Intravenous
Antibacterial	Vancomycin, erythromycin	Topical delivery
Anti-inflammatory	Prednisolone	Intravenous
Antifungal	Itraconazole	Topical delivery
Antivirus	Acyclovir, valacyclovir	Topical delivery
Gene therapy	DNA, siRNA	Intravenous
Antitumor	Doxorubicin, paclitaxel, doxorubicin, and cisplatin	Intravenous
Other	Curcumin, melatonin	Topical delivery/intravenous

## Data Availability

The data used to support the findings of this study are included within the article.
